The article "Predictors of depression among school adolescents in Northwest, Ethiopia, 2022: institutional based cross-sectional" was retracted in 2024. Reasons: content taken from a thesis; duplicated data; overlap with earlier publications; concerns about the data.

# Predictors of depression among school adolescents in Northwest, Ethiopia, 2022: institutional based cross-sectional

**DOI:** 10.1186/s12888-023-04899-2

**Published:** 2023-06-14

**Authors:** Aklile Tsega Chekol, Mastewal Aschale Wale, Agmas Wassie Abate, Eyerusalem Abebe Beo, Eman Ali Said, Berhan Tsegaye Negash

**Affiliations:** 1 Department of Nursing, College of Medicine and Health Sciences, Hawassa University, Hawassa, Ethiopia; 2 Department of Midwifery, College of Medicine and Health Sciences, Hawassa University, Hawassa, Ethiopia; 3 Department of Psychiatry, Dr. Ambachew Memorial Hospital, Amhara Regional Health Bureau, South Gondar, Ethiopia

**Keywords:** Northwest Ethiopia, High schools, Adolescents, Depression

## Abstract

**Background:**

Adolescent depression is a serious mental disorder that makes family problems, learning challenges, drug addiction, and increases absenteeism from school. It also has a major impact on a person’s ability to manage his or her daily tasks. In the end, the condition may result in self-destruction. Research is scarce among high schools in the study setting. Therefore, this study aimed to assess the prevalence and its associated factors of depression among high school adolescent students in Bahirdar City, Northwest Ethiopia in 2022.

**Methods:**

An institutional-based cross-sectional study was done from June 18 to July 16, 2022, among public and private high school adolescent students in Bahir Dar City, Amhara region, Ethiopia. A two-stage sampling technique was utilized. First, stratification by school type was made and schools were selected 30–40% by using a simple random sampling technique. Finally, an updated sampling frame was taken from each school director to select a sample of 584 study participants after proportional allocation by simple random sampling from six high schools. Patient Health Questionnaires were used to assess depression in high school students. The independent variables, like substance-related factors, were assessed by yes-or-no questions, and the academic stressor by academic stress in secondary education, was assessed by structured questionnaires. Binary and multivariate logistic regressions were used to identify factors associated with depression. Statistical significance was declared at a 95% confidence interval when the value of p was less than or equal to 0.05.

**Results:**

The response rate of the participants was 96.9%. The overall magnitude of adolescent depression was found to be 22.1% (95%CI 18.7, 25.7%). Being female (AOR: 3.43; 95%CI 2.11, 5.56), small family size (AOR: 3.01; 95%CI 1.47, 6.15); ever alcohol use (AOR: 2.40; 95%CI 1.51, 3.81); attending a public school (AOR: 3.01; 95%CI 1.68, 5.40), and having a history of abuse (AOR: 1.92; 95%CI 2.2, 3.08) were associated with depression.

The article "Predictors of depression among school adolescents in Northwest, Ethiopia, 2022: institutional based cross-sectional" was retracted in 2024. Reasons: content taken from a thesis; duplicated data; overlap with earlier publications; concerns about the data.

**Conclusion:**

In this study, the magnitude of depression among high school students in Bahir Dar City was higher than the national threshold. There was a significant association between sex, family size of parents, ever alcohol use, public schools, and having a history of abuse with depression among adolescents. Hence, it is better for schools to screen and provide intervention for depression in public high school students and offer therapies, especially in females and those with a history of abuse, small family size, or alcohol use.

## Background

Adolescence is an important period for the development of a socially integrated self-concept, while a negative self-concept may affect future decisions due to mental illness [1]. Approximately 20% of adolescents have some type of psychological disorder; of these, depression is the most common [2]. The period of adolescence represents a transitional stage from childhood to adulthood and represents the critical time frame during which an individual undergoes different developmental changes along with several emotional and psychosocial issues. Globally, it has been reported that depressive disorders often start at an early age, with rates ranging between 1 and 50% among adolescents [3]. Depression is a common psychiatric disorder that is characterized by a decrease in energy and interest, a feeling of guilt [4], difficulty concentrating, feelings of inferiority, and thoughts of death and suicide and is associated with a change in the level of activity, cognitive abilities, speech, sleep, appetite, and other biological rhythms [5]. Depression is a serious mental disorder among adolescents; as a result, it increases family problems, academic difficulties, substance abuse, and absenteeism. The problems can be either chronic or recurrent, which causes significant impairments in an individual’s ability to take care of his or her everyday tasks. At its worst, the illness causes self-destruction [6]. Among adolescents between the ages of 14 and 19, the magnitude was reported to range from 15 to 20% [7], and it is a global concern for children, adolescents, and adults even in developed nations [8].

According to the Depression Anxiety and Stress Scale (DASS), the magnitude of depression in Malaysia was 33.2% (21.5% moderate, 18.1% severe, and 3.0% extremely severe) [9], 34.5% in Qatar according to Beck’s Depression Inventory-II (BDI-II), [10], 39.7% in India according to the eleven-item Kutcher adolescent depression scale [7], 44.2% in Nepal according to the Epidemiologic Studies Depression Scale [11],45.9% in Kenya according to the Patient Health Questionnaire [12], 25% in Bangladesh according to the Epidemiological Studies Depression Scale (CESD-10) [13], and 36.2% in Aksum Ethiopia based on the Patient Health Questionnaire [14]. Suicidal thoughts, scholastic failure, poor relationships with family, friends, and other relatives, substance addiction, severe depression, and other mental co-morbidities are all caused by depression in adolescents [15]. The magnitude of depression among adolescents was high, ranging from 8 to 20% [16, 17]. In the world and India, respectively, adolescents experience emotional and behavioral issues that range from 16.5 to 40.8% and 13.7–50% [18–21]. Beginning at age 15, the annual incidence rates of depression in children and adolescents are 1–2% and 3–7%, respectively [22]. Around the ages of 12 for girls and 14 for boys, the prevalence rates start to rise. Among adolescents between the ages of 14 and 19 years old assessed on the Patient Health Questionnaire, the magnitude of depression was high at 8.4%, 12.6%, 15.4%, and 28%, respectively [23]. Around 48,910 children and adolescents died by suicide in 2010 as a result of depression, according to the CDC (2010) report. Males with depression are much more likely to succeed in committing suicide than females, even though females are more prone to attempt suicide. According to a systematic review of mental health issues in sub-Saharan adolescent populations, depression was 26.9% common [24]. Research is scarce in public and private high schools in the study setting. Therefore, this study aimed to assess the prevalence and its associated factors of depression among high school adolescents in public and private schools of Bahirdar City, Amhara region, Ethiopia in 2022.

The article "Predictors of depression among school adolescents in Northwest, Ethiopia, 2022: institutional based cross-sectional" was retracted in 2024. Reasons: content taken from a thesis; duplicated data; overlap with earlier publications; concerns about the data.

## Materials and methods

### Study design and setting

An institutional-based cross-sectional study design was conducted from June 18 to July 16, 2022, in Bahir Dar city high schools. The study was conducted among six high schools in Bahir Dar, a city in northwest Ethiopia. The city is situated at a distance of 490 km from Addis Ababa, the capital city of Ethiopia, and at an elevation of 1840 m above sea level. There was a total of 21 secondary schools in Bahir Dar, with a total of 26,504 students (10,916 male and 12,247 female), 1484 male students, and 1857 female students in 11 governmental high schools, and 10 privately owned high schools, respectively.

### Sample size determination and procedure

The sample size was calculated by single population proportion formula using the following assumptions; the proportion of depression was 36.2% among Ethiopia Aksum High School students [14], 95% confidence interval (1.96), 5% of margin error (0.05), and a design effect of 1.5. (n = Z_a/2_)^2^pq/d^2^. Plugging the value n= (1.96)^2^*0.36(1-0.36)/0.05^2^=354. Hence, we used multi-stage; we considered the stage and multiplied the sample size by a design effect of 1.5, and added a 10% non-response rate. A conservative design effect of 1.5 to cater for intra-cluster variability [25].

The article "Predictors of depression among school adolescents in Northwest, Ethiopia, 2022: institutional based cross-sectional" was retracted in 2024. Reasons: content taken from a thesis; duplicated data; overlap with earlier publications; concerns about the data.

The final calculated sample size was 584. Bahir Dar high school students were classified as either governmental or private. A two-stage sampling technique was utilized. First, stratification by school type was made and schools were selected 30–40% by using a simple random sampling technique after selecting three governmental and three private high schools using the simple random method as follows: grades nine, ten, eleven, and twelve. An updated sampling frame of students in each of the grade levels and sections was obtained from the academic director offices of each school. The framework included the name of students, sex, grade level, and sections, and data were obtained from the regional education office, the number total of students in **six** high schools during data collection was 10,387(grade nine = 3,531, grade ten = 2,588, grade eleven = 2,114, and grade twelve = 2,154). Then, a proportional allocation of study participants for each stratum (grade) was calculated. And the result was as follows: 225, 184,79,32,33, and 31 high school students (three from government and three from private) were selected from grades nine, ten, eleven, and twelve, respectively. Finally, a computer-generated lottery method was used to select study participants from each given grade level, resulting in the selection of 584 students (See Fig. 1).

**Fig. 1:** Variation of depression among school children between School types in Bahir-Dar city, Northwest Ethiopia, in 2022

### Operational definitions

#### Adolescents

Based on the World Health Organization age classification declared that adolescents aged 10–19 years [26].

#### Depression

Those who score great than or equal to 10 on the PHQ-9 scale [27].

#### Ever substance use

Those who had ever used substances (alcohol, chat, and cigarette) in their lifetime.

#### Current substance use

Those who have used substances (alcohol, chat, and cigarette) within the last 3 months.

#### Academic stress

measured using the Questionnaire of Academic Stress in Secondary Education (QASSE). The Questionnaire on Academic Stress in Secondary Education is designed to assess the wide variety of school sources and situations related to academic stress in adolescence. It comprises 30 items related to different potentially stress-producing situations in secondary education and it is measured on a 5-point Liker scale (1 = “Very low”, to 5 = “Very high”). It has internal consistency α = 0.89. A high mean score on the QASSE represents a high level of Academic stress [28].

The article "Predictors of depression among school adolescents in Northwest, Ethiopia, 2022: institutional based cross-sectional" was retracted in 2024. Reasons: content taken from a thesis; duplicated data; overlap with earlier publications; concerns about the data.

### Data collection tools

Data were collected by four psychiatric professionals using the Amharic language, (the national language of the country and the mother tongue of the students, by a semi-structured, self-administered questionnaire that has five parts: The first section includes participant socio-demographic characteristics such as age, sex grade, and so on; the second section assesses the outcome variable prevalence of depression using the Patient Health Questionnaire modified for adolescents (PHQ-9 A). The PHQ nine is a self-report instrument comprised of nine items with a four-point Likert scale, and the total score for each respondent was calculated by adding all nine items. Scores range from 0 to 27, and the sum of the nine items is categorized as follows: 0–4 minimal depression, 5–9 mild depression, 10–14 moderate depression, 15–19 moderately severe depression, and 20–27 severe depression [29]. Phq-9 for adolescents screening tool was validated in Ethiopia. The third part is academic-related factors, which were assessed through academic stress in secondary education. Structured yes/no questions were used to assess part four: clinical and psychological-related factors such as having a medical illness, a family history of mental illness, aggressive behavior, or a history of abuse. Finally, substance-related factors were assessed by a structured yes-or-no question.

### Data quality control

To control the quality of the data the questionnaire was prepared first in English and then translated to the Amharic language (the national language of the country) then it was translated back to English to ensure its consistency by language experts. The quality of data was also ensured through giving training for data collectors, supervision, and immediate reviewing of each of the completed questionnaires daily by the principal investigator and giving feedback the next morning for data collectors. The questionnaire was pretested one week before the actual data collection on 5% of the sample size (n = 29) outside the study area; the result is not included in the main study and the Cronbach alpha of the dependent variable assessment tool was 0.861. Based on the finding from the pretest, the final version of the questionnaire was established.

### Data processing and analysis

The collected data were checked for completeness, and consistency and then coded, all the completed data were entered using Epi-data version 4.6 and exported to Statistical Package for Social Science (SPSS) version 25 for analysis to generate descriptive statistics such as frequency, standard deviation, percentages, mean, and graph. The chi-square test was done before logistic regression to check its significance and necessary logistic regression assumptions were tested such as the normality test, multicollinearity, and Hosmer-Lemeshow model of fitness (0.533). After that logistic regression was used to identify an association between dependent and independent variables. A p-value cut-off 0.25 was used to reduce the number of variables entered in the regression model presuming that there would not be much change for the variables with p-value more than 0.25. In otherwords, to be more conservative for negative confounding and missing effective variables we considered a p-value of < 0.25 for entry. In multivariate logistic regression analysis, a p-value less than or equal to 0.05 and an adjusted odds ratio at a 95% CI were used to declare the statistical significance of the factors with the outcome variable.

The article "Predictors of depression among school adolescents in Northwest, Ethiopia, 2022: institutional based cross-sectional" was retracted in 2024. Reasons: content taken from a thesis; duplicated data; overlap with earlier publications; concerns about the data.

## Results

### Socio-demographic characteristics of study participants

Among the total number of 584 students invited to participate, 566 students completed the questionnaire, resulting in a response rate of 96.9%. However, only 3.1% of the study participants were non-respondents. In other words, these respondents did not complete any interviews. It was proved that their interruption is not related to depression. More than half of the participants were female students 302(53.4%). The average age of the students was 18.15 years, with a standard deviation of 1.295. Among those, 412 (74.6%) were found in the age group of 17–19 years. The majority of students follow an Orthodox Christian religion (See Table 1).

**Table 1:** Distribution of socio-demographic characteristics of the students in public and private high schools in Bahir Dar city, 2022 (n = 566)

Variables	Categories	Frequency	Percent
Sex	Male	264	46.6
	Female	302	53.4
Age	14–16	64	11.3
	17–19	422	74.6
	20–22	80	14.1
Religion	Orthodox	493	87.1
	Muslim	55	9.7
	Protestant	18	3.2
Grade level	9th	194	34.3
	10th	143	25.3
	11th	111	19.6
	12th	118	20.8
Family income in ETB	≤ 5000	272	48.1
	5001–7000	95	16.8
	> 7001	199	35.2
Occupations of parents	Government employee	178	31.4
	Merchant Farmer	282 106	49.8 18.7
Parent’s educational status	Unable to read and write	57	10
	Elementary school	257	47.2
	High school and above	242	42.8
Family size	1–3	`128	22.6
	4–6	378	66.8
	≥ 7	60	10.6

### Distribution of students

The maximum number of study participants in public schools were females (47.52%), while, the numbers of male and female students were almost similar in private schools (7.0%) (See Table 2). The distribution of grade levels from both public and private schools. The maximum numbers of students were in grades 9 and 10 from public and private schools, respectively (See Table 3).

The article "Predictors of depression among school adolescents in Northwest, Ethiopia, 2022: institutional based cross-sectional" was retracted in 2024. Reasons: content taken from a thesis; duplicated data; overlap with earlier publications; concerns about the data.

**Table 2:** Distribution of students in public and private schools (n = 566)

Sex	Public school	Private school	Total
Male	218	39	257
Female	269	40 (7.0%)	309
Total	487	79	566

**Table 3:** Showed grade level distribution of students in public and private schools (n = 566)

Grade level	Public school	Private school	Total
Grade 9	183	11	194
Grade 10	101	42	143
Grade 11	103	8	111
Grade 12	100	18	118
Total	487	79	566

### Substance-related factors

From the total number of students, 52 (9.2%) have chewed chat in their lifetimes, and 47 (8.3%) have chewed chat within the last 3 months. Whereas 315 (55.7%) of students had consumed alcohol in their lifetime, 210 (37.1%) had consumed alcohol in the previous three months. Regarding cigarette smoking, 36 (6.4%) of students smoke cigarettes in their lifetime, and 30 (5.3%) smoke cigarettes within the last three months (See Table 4).

**Table 4:** Description of substance use among school adolescents in public and private students in Bahir Dar city, 2022 (n = 566)

Variables	Categories	Response	Frequency	Percent
Ever substance use	Khat	Yes	52	9.2
		No	514	90.8
	Alcohol	Yes	315	55.7
		No	251	44.3
	Tobacco	Yes	36	6.4
		No	530	93.6
Current substance use	Khat	Yes	47	8.3
		No	519	91.7
	Alcohol	Yes	210	37.1
		No	356	62.9
	Tobacco	Yes	30	5.3
		No	536	94.7

### Clinical and psychological-related factors

Of the total number of students, 146 (25.7%) had medical illnesses. Likewise, 66 (11.7%) had a family history of mental illness, and 130 (23.0%) had experienced abuse in their lifetime. Regarding aggressive behavior, 18.4% and 12.95% have physical and verbal aggression, respectively.

### Academic-related factors

The mean of the academic stressor questions is 80.28 with an SD of 19.66. Of the total students, 303 (53.5%) had values above the mean and were categorized as having academic stressors, while the remaining 263 (46.5) had values below the mean.

### The magnitude of depression

In this study, the magnitude of depression in adolescents was found to be 125 (22.1%) with (95% CI of 18.7, 25.7%). Of those, 27.2% and 72.8% were from private and public schools, respectively. According to Fig. 2 report, 69(12.2%) participants experienced moderate depression, 51 (9%) experienced moderately severe depression, and 5 (0.9%) experienced severe depression (See Fig. 2).

**Fig. 2:** Schematic representation of the sampling procedure

### Associated factors of depression

Sex, age, residence, family size of parents, income, history of alcohol use, aggressive behavior, school type, and having a history of abuse were found to have P-values less than 0.25 in binary logistic regression and be candidates for multiple logistic regressions. However, in the multiple logistic regressions, sex, family size of parents, alcohol use, public school, and having a history of abuse were significantly associated with depression in adolescents’ depression.

The article "Predictors of depression among school adolescents in Northwest, Ethiopia, 2022: institutional based cross-sectional" was retracted in 2024. Reasons: content taken from a thesis; duplicated data; overlap with earlier publications; concerns about the data.

The odds of developing depression in adolescence were threefold higher in female students as compared to male students (AOR = 3.43; 95% CI: 2.11, 5.56). In this finding, the odds of developing depression among parents who have a small family size are threefold higher as compared to parents who have a large family size (AOR = 3.01; 95% CI = 1.47,6.15). The odds of depression among students who have ever used alcohol were two times higher as compared to those who did not drink (AOR = 2.40; 95% CI 1.51,3.81). The odds of developing depression among students who attend their education at public schools were threefold higher as compared to students who attend their education at private schools (AOR = 3.01; 95%CI 1.68, 5.40) and the odds of developing depression among students who have a history of abuse was two times higher as compared to students who have no abuse history (AOR = 1.92; 95%CI 2.20, 3.08) (See Table 5).

**Table 5:** Bivariate and Multivariate logistic regression analysis of depression and associated factors among public and private high school students at Bahir Dar city, 2022 (n = 566)

Variables	Categories	Depression		COR (95% CI)	AOR (95% CI)	p-value
		Yes	No			
**Sex**	Male	34	223	1	1	
	**Female**	**91**	**218**	0.65 (0.24, 0.57) *	3.43(2.11,5.56) **	**0.001**
Age	14–16	23	72	1.05(0.52, 2.12)	1.49(0.67, 3.34)	0. 331
	17–19	84	310	0.89 (0. 50, 1.59)	1.16 (0.61, 2.19)	0. 0.654
	20–22	18	59	1	1	
Residence	Rural	19	66	3.01(1.65, 5.49)	1.26(0.66, 2.37)	0. 485
	Urban	42	439	1	1	
**Family size**	**1–3**	**45**	**86**	3.63 (1.89, 6.95) *	3.01 (1.47,6.15) **	**0.003**
	**4–6**	**65**	**251**	1.80(0.98, 3.29) *	2.07 (1.08,3.97) **	**0.028**
	≥ 7	15	104	1	1	
Average monthly income of family	< 5000	69	203	1.50(0.71, 3.13)	1.96(0.87, 4.4 6)	0.416
	5001 − 700	18	77	1.03(0. 44, 2.42)	0 0.45 (0.12, 1.89)	0. 27
	7001–10,000	28	117	1.05(0.47, 2.35)	1.46 (0.46, 4.62)	0.519
	≥ 10,000	10	44	1	1	
**Ever alcohol use**	Yes	**54**	**258**	0.54 (0.36, 0.81) *	2.40 (1.51,3.81) **	**< 0.001**
	No	71	183	1	1	
**School type**	**Public**	**91**	**396**	0.30 (0.28,0 0.83) *	3.01 (1.68, 5.40) **	**< 0. 001**
	Private	34	45	1	1	
**History of abuse**	**Yes**	**50**	**111**	1.98(1.31, 3.01) *	1.92(2.20,3.08) **	**0. 007**
Aggressive behaviors	No	75	330	1	1	
	Yes	28	76	1.39(0.85, 2.26)	0.58 (0.32, 1.06)	0.075
	No	97	365	1	1	

Key; *P-value < 0.025; **P-value < 0.05; 1 = Reference group; OR = Adjusted Odds Ratio; COR = Crude Odds Ratio

The article "Predictors of depression among school adolescents in Northwest, Ethiopia, 2022: institutional based cross-sectional" was retracted in 2024. Reasons: content taken from a thesis; duplicated data; overlap with earlier publications; concerns about the data.

## Discussion

The current study showed that the magnitude of depression among high school adolescent students was 22.1% (95%CI 18.7–25.7%). This finding is in line with the finding of a study conducted in Uganda (21.0%) [30], Malaysia (21.41%) [31], Korea (20.6%) [32], Nigeria (21.2%) [33], China (19.9%) [34], and in India (20.3%) [35]. The reason for the agreement could be similar screening tools used in both the previous and present studies which were patient health questionnaires. Moreover, the other possible reason for their similarity could be using the same study populations in the previous and current studies.

This finding was higher than the findings of studies conducted in Malaysia (10.3%) [36], Nigeria (16.3%) [37], Thailand (14.19%) [38], Korea (13.6%) [39], and Jamaica (14.2%) [40]. On the other hand, the finding of this study was lower than study finding conducted in Nepal (44.2%) [11], Qatar (34.5%) [10], Iran (37%) [41], India (39.7%) [7], Turkey (45.1%) [42], Kenya 45.9% [12], Bangladesh (25%) [13], and Aksum town Ethiopia (36.2%) [14]. The reason for the above difference might be due to the difference in screening tool which was a structured self-administered questionnaire developed from the Goldberg Depression Questionnaire in Nigeria [43], and the children’s depression inventory in a study in Malaysia [36], in Turkey BDI, in India, eleven item Kutcher adolescent depression scale were utilized, in Qatar BDI-II was used, in Bangladesh Epidemiological Studies Depression Scale (CESD-10) was used. The other possible variation might be due to sample size variations. Moreover, the discrepancy might be due to cultural variation across different nations.

The results of this study showed that female students had higher levels of depression than male pupils. This result is consistent with research that was done in other counties [7, 10, 41–43]. The reason for this discrepancy may be related to how the symptom manifests itself. Males typically exhibit externalizing symptoms, but females frequently exhibit internalizing problems [44]. There are particular types of depression-related sickness that affect women only, such as premenstrual dysphoric disorder, postpartum depression, and postmenopausal depression and anxiety, which are linked to changes in ovarian hormones and may explain the rise in female sufferers. Because men and women have different numbers of chromosomes—women have two copies of the X chromosome and men have one—the depression rate varies by gender. As a result, sexual disparities in the propensity for mental diseases are conferred by genetic variances. Despite this intricacy, recent research revealed that biological variables, such as change in ovarian hormone levels, and decreasing estrogen in particular, may contribute to women’s depression [45]. Further, other potential causes for this gender difference have been identified, including biological, genetic, psychological, hormonal, and family influences. depression [43].

The article "Predictors of depression among school adolescents in Northwest, Ethiopia, 2022: institutional based cross-sectional" was retracted in 2024. Reasons: content taken from a thesis; duplicated data; overlap with earlier publications; concerns about the data.

Attending education in public schools contributes to the development of depression among high school students. The current study reported that participants who attended public school had more depression than those who attended private schools. This finding was supported by a study conducted on the magnitude and factors associated with depression among school-going adolescents in Chandigarh, North India. This difference can be explained by the socioeconomic difference between the students of the two types of schools [35].

In this study, abuse history is another associated factor that contributes to the development of depression among high school students. Students who have an abuse history had more than twofold of having depression than those who have no history of abuse. The finding is supported by a study done UK Biobank [46]. Experiences of childhood sexual/physical abuse may lead to feelings of entrapment, habituation to pain, and reduced fear of death which may result in a greater capacity for suicidal behavior as a means of escape [47]. A recent study has suggested that adverse social relationships during childhood can also contribute to depressive symptoms including suicidal behavior [48].

Another element that influences the onset of depression is the size of the family. According to recent studies, smaller families tend to have more depressed members than bigger families. Big families typically provide for their members on a social, emotional, and financial level. Students from large homes typically have more social duties than kids from small families, which explains why. [49]. Reduced household size has a number of socioeconomic and health effects such as poor mental health and depression. [50–52]. Those with small families tend to experience depression more frequently than those with large families, on average. [53], This proposes that individuals living in little family units are more likely to endure misery than those living in expansive families [54]. Unfavorable well-being impacts such as sadness are known to be relieved by family bolster. This incorporates enthusiasm, fabric, and other unmistakable bolster components that act as buffers against mental and other afflictions by lessening powerlessness to well-being and social stuns [55]. This result is due to family caregiving, a defensive figure against social stun [55]. As more people marry, have children, and join common families, larger households form. Members can exchange experiences, create new memories, get help on the emotional and financial fronts, and broaden their social circles during these gatherings. Sharing responsibilities, meals, and costs benefits one’s mental health and lowers the risk of developing depression. Children from large families interact with one another more than kids from smaller households, which may indicate that they learn social skills like collaboration and sharing early [49]. This result, however, conflicts with a study carried out in southwest Nigeria, which revealed a strong correlation between the prevalence of depression and the number of adolescent siblings. This is due to the fact that each child in a big household receives less attention and resources. Another explanation is that the high density of families in polygamous environments makes it difficult for parents to provide for their offspring as they develop love, nurturing, assistance from parents, emotional support, and financial need [43].

The article "Predictors of depression among school adolescents in Northwest, Ethiopia, 2022: institutional based cross-sectional" was retracted in 2024. Reasons: content taken from a thesis; duplicated data; overlap with earlier publications; concerns about the data.

And, finally, alcohol use contributed to the development of depression. In the current finding, students who drink alcohol experience higher depression than those who don’t. This is supported by a study finding from Malaysia which revealed that increased alcohol use was associated with an increase in the lifetime occurrence of depressive disorders in adolescents, and the rates of psychiatric co-morbid were highest in adolescents with problematic alcohol use [56]. The rates of major depressive disorder and alcohol use disorder were low in adolescence (2%), but increased in early adulthood (11%) and adulthood (7%), indicating that the problem of alcohol use in adolescence predicts early adult major depressive disorder [57]. However, there is a bi-directional association between the two, meaning that alcohol use disorder can cause depression to worsen and vice versa. Because of this, the study is cross-sectional and requires further longitudinal research by the researcher in the future.

### Strengths and limitations of the study

The study includes a large sample size from governmental and private schools, which makes it more generalizability, using validated tools. On the other hand, the limitations of the study; social desirability bias could be affecting the finding due to sensitive questions related to substance use, being a cross-sectional study design was the other limitation hence, it did not show the causal effect relationship. Peer influence was not assessed.

The article "Predictors of depression among school adolescents in Northwest, Ethiopia, 2022: institutional based cross-sectional" was retracted in 2024. Reasons: content taken from a thesis; duplicated data; overlap with earlier publications; concerns about the data.

## Conclusion

The magnitudes of depression in Bahir Dar City among high school adolescent students are found to be higher than the national threshold. There was a statistically significant association between sex, small family size, ever alcohol use, public schools, and having a history of abuse with adolescents’ depression.

### Clinical and public implications

Better to initiate school-based mental health services in schools and conduct regular mental health screenings, and provide appropriate interventions by the regional health bureau, especially for female students. It is better for schools to screen and provide intervention for depression in public high school students and offer therapies, especially in females and those with a history of abuse, small family size, or alcohol use. For the benefit of upcoming researchers, it would be better to conduct a prospective cohort study to ascertain the origins, effects, and contributing elements of depression. By integrating the system in schools, stakeholders had a responsibility to emphasize the value of routine mental health screenings and early intervention.

## Data Availability

The data is available upon request by the corresponding author.
